# Essential Oils Loaded in Nanosystems: A Developing Strategy for a Successful Therapeutic Approach

This article has been retracted.

**DOI:** 10.1155/2014/651593

**Published:** 2014-05-29

**Authors:** Anna Rita Bilia, Clizia Guccione, Benedetta Isacchi, Chiara Righeschi, Fabio Firenzuoli, Maria Camilla Bergonzi

**Affiliations:** ^1^Department of Chemistry, University of Florence, Via U. Schiff 6, 50019 Sesto Fiorentino, Italy; ^2^Center for Integrative Medicine, Careggi University Hospital, University of Florence, 50124 Florence, Italy

## Abstract

Essential oils are complex blends of a variety of volatile molecules such as terpenoids, phenol-derived aromatic components, and aliphatic components having a strong interest in pharmaceutical, sanitary, cosmetic, agricultural, and food industries. Since the middle ages, essential oils have been widely used for bactericidal, virucidal, fungicidal, antiparasitical, insecticidal, and other medicinal properties such as analgesic, sedative, anti-inflammatory, spasmolytic, and locally anaesthetic remedies. In this review their nanoencapsulation in drug delivery systems has been proposed for their capability of decreasing volatility, improving the stability, water solubility, and efficacy of essential oil-based formulations, by maintenance of therapeutic efficacy. Two categories of nanocarriers can be proposed: polymeric nanoparticulate formulations, extensively studied with significant improvement of the essential oil antimicrobial activity, and lipid carriers, including liposomes, solid lipid nanoparticles, nanostructured lipid particles, and nano- and microemulsions. Furthermore, molecular complexes such as cyclodextrin inclusion complexes also represent a valid strategy to increase water solubility and stability and bioavailability and decrease volatility of essential oils.

## 1. Introduction

Spices have been used since antiquity for their perfume, medicinal and preservative properties and to impart aroma and flavour to food. Hippocrates, the “father of medicine,” prescribed perfume fumigations and massages with aromatic oils. Turpentine was known by the Greeks and Romans for its properties against lung diseases and biliary lithiasis. Dioscorides saying the best was the white, clear variety. Pliny, Hippocrates, and Galen favoured its properties too. Venice turpentine was known during the Middle Ages, and the city became one of the principal markets for this medicinal drug [1]. The first distillation of essential oils appeared in the East (India and Persia) [1] more than 2000 years ago and was improved in the 9th century by the Arabs [2]. Nevertheless, the first authentic written account of distillation of essential oil is ascribed to Villanova (ca. 1235–1311), a Catalan physician [1], and only by the 13th century, the essential oils (EOs) were being made by pharmacies and their pharmacological effects were described in pharmacopoeias [2]. By contrast, their use does not appear to have been widespread in Europe until the 16th century; turpentine, juniper wood, rosemary, spike (lavender), clove, mace, nutmeg, anise, and cinnamon became common essential oils. In this century the term “essential oil” was used for the first time by Paracelsus von Hohenheim, who named the effective component of a drug, “Quinta essential” [1]. By the middle of the 20th century, the role of essential oils had been reduced almost entirely to be used in perfumes, cosmetics, and food flavourings: rather in pharmaceutical preparations they still represent an important part of the traditional medicine and several monographs are reported in the official pharmacopoeias. At present ca. 3000 essential oils (EOs) are known, and 10% of them have commercial importance [3] for the pharmaceutical, agronomic, food, sanitary, cosmetic, and perfume industries.

## 2. EOs Chemical Composition

EOs are volatile, limpid, and rarely coloured liquids, lipid soluble and soluble in organic solvents with a generally lower density than that of water. They can be synthesized by all plant organs, that is, buds, flowers, leaves, stems, twigs, seeds, fruits, roots, wood, or bark and are stored in secretory cells, cavities, canals, epidermic cells, or glandular trichomes. Constituents are lipophilic and highly volatile secondary plant metabolites, reaching a mass below a molecular weight of 300, that can be physically separated from other plant components or membranous tissue [4].

Nowadays there are several methods for extracting essential oils. These may include use of liquid carbon dioxide or microwaves, low or high pressure distillation employing boiling water or hot steam. As defined by the International Organization for Standardization (ISO), the term “essential oil” is reserved for a “product obtained from vegetable raw material, either by distillation with water or steam, or from the epicarp of citrus fruits by a mechanical process, or by dry distillation” (ISO 9235, 1997), that is, by physical means only. Furthermore, essential oils for medical purposes need to comply with national or international pharmacopoeias.

The chemical profile of the essential oil products differs not only in the number and type of molecules but also in their stereochemical structures, and can be very different according to the selected method of extraction. The extraction product can fluctuate in quality, quantity, and composition according to climate, soil composition, plant organ, age, and vegetative cycle stage [5]. Most of the commercialized essential oils are chemotyped by gas chromatography and mass spectrometry analysis. Analytical monographs have been published (European Pharmacopoeia, ISO, WHO, Council of Europe) to ensure good quality of essential oils. The EOs are generally complex mixtures of volatile organic compounds produced as secondary metabolites in plants; they include hydrocarbons (terpenes and sesquiterpenes) and oxygenated compounds (alcohols, esters, ethers, aldehydes, ketones, lactones, phenols, and phenol ethers) [1].

Generally EOs contain about 20–60 components up to more than 100 single substances, at quite different concentrations; two or three are major components at fairly high concentrations (20–70%) compared to others components present in trace amounts. For example, carvacrol (30%) and thymol (27%) are the major components of the* Origanum* species essential oil.

Generally, these major components determine the biological properties of the essential oils. The components include different groups of distinct biosynthetical origin. The main group is composed of terpenoids, phenylpropanoids, and short-chain aliphatic hydrocarbon derivatives, which are all characterized by low molecular weight. Representative structures are depicted in Figure 1.

Terpenes are made from combinations of several 5-carbon-base (C5) units called isoprene and form structurally and functionally different classes. The biosynthesis of the terpenes consists of synthesis of the isopentenyl diphosphate (IPP) precursor, repetitive addition of IPPs to form the prenyldiphosphate precursor of the various classes of terpenes, modification of the allylic prenyldiphosphate by terpene specific synthetases to form the terpene skeleton, and, finally, secondary enzymatic modification (redox reaction) of the skeleton to attribute functional properties to the different terpenes. Terpenoids derive from the C5-building blocks isopentenyl diphosphate (IPP) and its isomer dimethylallyl diphosphate (DMAPP) and are generally represented by monoterpenes (C10) and sesquiterpenes (C15), while hemiterpenes (C5) are quite rare [6]. Terpenes containing oxygen in the form of hydroxyl, ether, aldehyde, ketone, or carboxylic moieties are called terpenoids.

The monoterpenes (Figure 1) are formed from the coupling of two isoprene units (C10). They are the most representative molecules constituting 90% of the essential oils and allow a great variety of structures. They consist of several functions including acyclic hydrocarbons (myrcene and ocimene); monocyclic hydrocarbons (limonene, terpinenes, p-cymene, and phellandrenes); bicyclic hydrocarbons (pinenes, camphene, and sabinene); acyclic alcohols (geraniol, linalool, citronellol, lavandulol, and nerol); monocyclic alcohols (menthol, *α*-terpineol, and carveol); bicyclic alcohols (borneol, fenchol, chrysanthenol, and thuyan-3-ol); acyclic aldehydes (geranial, neral, and citronellal); acyclic ketone (tegetone), monocyclic ketone (menthones, carvone, pulegone, and piperitone); bicyclic ketone (camphor, fenchone, thuyone, and pinocarvone); acyclic esters (linalyl acetate or propionate and citronellyl acetate); monocyclic esters (menthyl or *α*-terpinyl acetate); bicyclic esters (isobornyl acetate); ethers (1,8-cineole and menthofuran); peroxides (ascaridole); and phenols (thymol, carvacrol).

The sesquiterpenes are formed from the assembly of three isoprene units (C15). The extension of the chain increases the number of cyclisations which allows a great variety of structures (Figure 1). Also sesquiterpenes include hydrocarbons (azulene, *β*-bisabolene, cadinenes, *β*-caryophyllene, farnesenes, and zingiberene); alcohols (bisabolol, *β*-nerolidol, farnesol, *β*-santalol, and patchoulol); ketones (germacrone, *β*-vetinone, and turmerones); and epoxide (caryophyllene oxide and humulene epoxides).

Other aromatic molecules are phenylpropanoids formed via the shikimic acid pathway leading to phenylalanine [6] and occurring less frequently than the terpenes.

Aromatic compounds originated from the shikimate pathway (phenylpropanoids, Figure 1) comprise aldehydes (cinnamaldehyde); alcohols (cinnamic alcohol); phenols (chavicol and eugenol); methoxy derivatives (anethole, estragole, and methyleugenols); methylenedioxy compounds (apiole, myristicin, and safrole).

Nitrogenous or sulphured components such as glucosinolates or isothiocyanate derivatives (garlic and mustard oils) are also characteristic secondary metabolites of diverse aromatic plants or of processed, grilled, or roasted products. In addition, some essential oils contain photoactive molecules like coumarins and furocoumarins (*Citrus aurantium* ssp.* bergamia* essential oil contains psoralens) and short-chain aliphatic substances such as 3-octanone and methyl nonyl ketone (Figure 1).

## 3. Limits and Challenges for the Rational Clinical Use of Essential Oils

The most recent applications of EOs include being as antioxidants and preservatives in food [7], incorporated into foodstuff packaging material [8], and application as plant and crop protectants [9]. Traditionally, essential oils have been used for many biological properties including bactericidal, virucidal, fungicidal, antiparasitical, insecticidal, and other medicinal properties such as analgesic, sedative, anti-inflammatory, spasmolytic, and locally anesthetic remedies [9–11].

At present, promising approaches have been reported using essential oils or components thereof in medicinal products for human or veterinary use [12]. The most effective way to use most EOs is by external application, as gargles and mouthwashes or inhalation; rarely they are used orally even if generally regarded as safe (GRAS) to ingest. In this case of oral administration they are generally diluted with milk, soy milk, or olive oil. Topical application is generally safe; the oil is diluted in a formulation but sometimes can give skin reactions and in particular some oils (specifically citrus oils) are UV sensitive and may cause irritation or darkening of skin upon exposure to sunlight up to 4 days after application.

In case of inhalation when using strong oils, limit time in immediate vicinity of an essential oil diffuser as the concentrated vapours may cause eye irritation, some of them are not recommended for diffusing or direct inhalation.

There is adequate evidence suggesting that although essential oils are metabolized quickly, their distribution throughout the body is considered to be relatively high.

Most essential oil components are metabolized and either eliminated by the kidneys in the form of polar compounds following limited phase I enzyme metabolism by conjugation with glucuronate or sulfate or exhaled via the lungs as CO_2_. For example, after oral administration of (−)-menthol, 35% of the original menthol content was excreted renally as menthol glucuronide [13, 14]. The same happens with thymol, carvacrol, limonene, and eugenol. After their oral administration, sulphate and glucuronide forms have been detected in urine and in plasma, respectively [15, 16]. The fast metabolism and short half-life of active compounds have led to the belief that there is a minimum risk of accumulation in body tissues [17].

EO compounds are small, fat soluble molecules, able to permeate the membranes including the skin before being captured by the microcirculation and drained into the systemic circulation, which reaches all targets organs [9, 18]. In general, the respiratory tract offers the most rapid way of entry followed by the dermal pathway [19]. Topically, aromatherapy EOs can sometimes cause irritation of the skin, especially if the oils are not diluted. Some oils, such as bergamot oil, can also cause photosensitization and induce malignant change. Applying excessive amounts of highly concentrated oils to a large surface of the skin or on broken skin can result in significant systemic absorption and increase the chance of serious side effects, such as convulsions because EOs are permeation enhancers.

Besides the high volatility, EOs can easily decompose, owing to direct exposure to heat, humidity, light, or oxygen. A recent manuscript has reviewed the factors influencing essential oil stability; specific knowledge on the chemical composition and properties of essential oil is fundamental for an adequate use [20].

Degradation of EOs constituents is due to oxidation, isomerization, cyclization, or dehydrogenation reactions, triggered either enzymatically or chemically [21], strongly influenced by the conditions during processing and storage of the plant material, upon distillation, and in the course of subsequent handling of the oil itself [22]. Furthermore, besides organoleptic alterations and viscosity changes, some aged essential oils as well as oxidized terpenoids have revealed skin-sensitizing capacities [23] leading to a hypersensitivity reaction synonymous to allergic contact dermatitis [24].

## 4. Nanoencapsulation Technology

Encapsulation of bioactive compounds represents a feasible and efficient approach to modulate drug release, increase the physical stability of the active substances, protect them from the interactions with the environment, decrease their volatility, enhance their bioactivity, reduce toxicity, and improve patient compliance and convenience [25].

A significantly large part of current literature on the encapsulation of EOs deals with micrometric size capsules, which are used for the protection of the active compounds against environmental factors (e.g., oxygen, light, moisture, and pH), to decrease oil volatility and to transform the oil into a powder. Encapsulation in nanometric particles is an alternative for overcoming these problems but additionally, due to the subcellular size, may increase the cellular absorption mechanisms and increasing bioefficacy.

Nanosystems applied to the skin are used to facilitate local therapies even if it is still under discussion of the mechanisms of penetration trough skin. It is accepted that topical drug delivery with nanoparticles targets the nanoparticles into the deeper layers of skin and generally they do not reach the viable epidermis. Only where the cheratine barrier is compromised, however, such as in aged or diseased skin, an enhanced particle penetration occurs. The use of nanoparticles provides a sustained and slow release of the active constituents; nanoparticles represent a reservoir. In addition, nanoparticles can interact with skin at a cellular level as adjuvants to enhance immune reactivity for topical vaccine applications.

Hair follicles and furrows were regarded as insignificant as potential routes for drug delivery, covering less than 1% of the human skin surface area, but their complex vascularisation and deep invagination with a thinning stratum corneum have led to a reappraisal of this view. It has been demonstrated that in particular hair follicles are an efficient reservoir for nanoparticle-based drug delivery and nanoparticles penetration can be increased with massage [26, 27].  Figure 2 shows that the potential sites for skin targeting nanoparticles include the surface of the skin, furrows, and hair follicles.

The alternative routes of administration of EOs are represented by oral intake and inhalation.

Within these routes the nanodelivery systems encounter the mucosal lining of the nasal, lung, oral (sublingual and buccal) cavity, stomach, and gut. Nanocarriers can improve the stability of EOs against enzymatic degradation, achieve desired therapeutic levels in target tissues for the required duration with a lower number of doses, and might ensure an optimal pharmacokinetic profile to meet specific needs. However, the viscous, elastic, and sticky mucus layer that lines all mucosa tissues (even if with different characteristics) has evolved to protect the body by rapidly trapping and removing foreign particles and hydrophobic molecules. As a consequence, mucoadhesion defined as the ability of nanoparticle to adhere to the mucus enhancing drug absorption can represent a valid strategy to enhance the residence time of the nanosystem and enhance absorption and bioavailability of the active constituent because it can facilitate transport across the epithelium. The interaction is generally achieved with natural or synthetic polymers which can form hydrogen bonding and hydrophobic or electrostatic interactions with mucin. The electrostatic interaction is the most effective and it can be achieved using positively charged polymers such as chitosan, being mucin negatively charged [28–32].

Particle size, shape, and surface properties of the nanoparticles play a crucial role in the uptake of nanosized delivery systems across the mucosal membrane. The nanocarriers with particle size of 50–300 nm, positive zeta potential, and hydrophobic surface were found to have preferential uptake as compared to their counterparts [28].

Diverse absorption mechanisms have been established and two have been predominantly used: the paracellular route that is slow and passive and the transport through a lipoidal route and it is also known as the transcellular process which is responsible for the transport of lipophilic drugs that show a rate dependency on their lipophilicity. Drug also crosses cell membranes by an active transport route via carrier-mediated means or transports through the opening of tight junctions interacting with the tight junction proteins [28–32].

For instance the increase in the absorption of nanocarriers by enterocytes is due to tight junction modulation, receptor-mediated endocytosis and transcytosis, phagocytosis via specialized microfold cells (M cells) of the Peyer's patches, and other mucosa associated lymphoid tissues (MALT) and lymphatic absorption via chylomicron uptake mechanism from the enterocytes (mediated by lipase for various lipid-based drug delivery systems) [29]. Mechanism of carriers penetration through enteric mucosa is reported in Figure 3.

## 5. EO-Loaded Nanodelivery Systems

Nanodelivery systems can be engineered to possess a number of desirable features for therapy, including (i) sustained and controlled release of drugs locally, (ii) deep tissue penetration due to the nanometric size, (iii) cellular uptake and subcellular trafficking, and (iv) protection of cargo therapeutics at both extracellular and intracellular levels.

Nanocarriers can be structured by a great variety of material and designs. This review is focused on the organic nanocarrier systems, characterised by high biodegradability and biocompatibility, and classified in polymer-based nanoparticles and lipid-based nanoparticles. In addition molecular complexes such as inclusion complexes with cyclodextrins are reported. A schematic representation of nanosystem platforms for EOs is reported in Figure 4.

### 5.1. Polymer-Based Nanocarriers

Polymeric nanocarriers are classified as nanocapsules and nanospheres. Nanocapsules have two compartments: a polymeric wall and a core, which is commonly oily. Nanospheres are matrix systems. The essential oil may be conjugated with the polymer (matrix or wall) or in the oily core.

Biocompatible polymers of synthetic origin include poly-*α*-cyanoacrylate alkyl esters, polyvinyl alcohol, polylactic acid, polyglycolic acid, and polylactic glycolic acid. The latter is usually divided into two classes: polysaccharides and proteins. Polysaccharides include compounds from plant origin (e.g., pectin, cellulose and its derivatives, starch and its derivatives, arabic gum, carrageenan, and alginate) and polysaccharides from microbial or animal origin (e.g., xanthan gum and chitosan). Proteins are albumin, gelatine, soy proteins, and casein. Nanoparticles made of polysaccharides, due to their unique properties, are promising carriers to deliver and protect the physiological properties of hydrophilic drugs and have been successfully applied as drug delivery systems [33]. As natural biomaterials, polysaccharides are stable, safe, nontoxic, hydrophilic, and biodegradable. In addition, polysaccharides have abundant resources in nature and low cost in their processing. The release of EOs from carriers occurs through one of the following processes: dissolution, desorption of the surface-bound/adsorbed functional ingredient, diffusion through the matrix; matrix erosion including enzyme degradation, and a combination of these processes [34].

Eugenol represents the main constituents of diverse EOs but it is highly volatile, unstable, and sensitive to oxygen, light, and heat during processing, utilization, and storage. Choi et al. [35] reported that encapsulation of eugenol into polycaprolactone nanoparticles could enhance its stability against light oxidation.

Eugenol has been also encapsulated into chitosan nanoparticles with an average size of less than 100 nm. Loading capacity was 12% and encapsulation efficiency was 20%. The particles had positively charged surface, with a zeta potential value ranging from +16.2 to +33.5 mV. The eugenol-loaded chitosan nanoparticles were thermally stable and could be useful as antioxidants for various thermal processing applications [36].

Chitosan nanoparticles have also been developed with oregano essential oil known for its potent antioxidant and antimicrobial activity. The obtained nanoparticles exhibited a regular distribution and spherical shape with size range of 40–80 nm and the encapsulation efficiency and loading capacity were about 21–47% and 3–8%, respectively, when the initial EO content was 0.1–0.8 g/g chitosan.* In vitro* release studies showed an initial burst effect and followed by a slow drug release [37].

Alginate/cashew gum nanoparticles were prepared via spray-drying to encapsulate* Lippia sidoides* essential oil, rich in thymol which has fungicide and bactericide activities. Cashew gum is a biopolymer extracted from the exudate of* Anacardium occidentale*, a common tree of Brazil's Northeastern region. The gum main chain is composed of galactose (72%), with side-chains of arabinose (4.6%), glucose (14%), rhamnose (3.2%), and uronic acid (4.7%). The averaged sizes of the nanoparticles were in the range 223–399 nm, and zeta potential values ranging from −30 to −36 mV. Encapsulated oil levels varied from 1.9 to 4.4% with an encapsulation efficiency of up to 55%. The* in vitro* release profile showed that between 45 and 95% of oil was released within 30–50 h. The addition of cashew gum to alginate has proven to be able to maximize the hydrophilic character of the polymer matrices, allowing a quicker release at a satisfactory oil loading. Moreover, the oil release profile revealed that the use of alginate in synergy with cashew gum for EO encapsulation presents itself as a potential delivery system with tailored release rate, loading, and encapsulation efficacy [38].

Using the same EO from* Lippia sidoides* nanoparticles made of chitosan (a deacetylated form of chitin, chemically D-glucosamine and N-acetyl-D-glucosamine linked by beta (1–4) linkages) and cashew gum aimed to improve essential oil loading and release profiles. Samples designed using relative ratios, matrix: oil, 10 : 2; gum : chitosan, 1 : 1; and 5% gum concentration, showed high loading (11.8%) and encapsulation efficiency (70%), with average sizes in the range 335–558 nm.* In vitro* release profiles showed that nanoparticles presented slower and sustained release. The nanocarriers presented efficacy against* St. aegypti* larvae, where the mortality rate was related to the loading values and gum : chitosan ratios. In particular, samples gum : chitosan 1 : 1 and gum : chitosan 1 : 10 showed, respectively, 87% and 75% of mortality after 48 h, reaching over 90% of mortality at 72 h. These results showed that the gum-chitosan nanoparticles were designed and present sustained release features [39].

The formation of heat-resistant flavour nanocapsules of jasmine essential oil was achieved by gelatin and arabic gum. Their heat-resistance capability against 80°C was evaluated by both structural characteristics (size, polydispersity index, and zeta potential) and flavour analysis. The results showed that the nanocapsules were stable at 80°C for 7 h, even if the GC-MS revealed that jasmine essential oil began to destroy above 5 h [40].

Thymol loaded in zein (a corn prolamine protein) nanoparticles stabilized with sodium caseinate and chitosan hydrochloride were prepared and characterized. In the absence of sodium caseinate, the particle size and zeta potential of zein nanoparticles were 118.30 nm and +28.10 mV, respectively. The zeta potential of rein nanoparticles after coating with sodium caseinate reversed from positive to negative (in the range of −33.60 to −38.95 mV), while size was around 200 nm. Due to the presence of sodium caseinate, the stabilized zein nanoparticles showed a shift of isoelectric point from 6.18 to 5.05 and had a desirable redispersibility in water at neutral pH after lyophilization. Encapsulated thymol was more effective in suppressing Gram-positive bacterium than unencapsulated thymol for a longer time period. Zein nanoparticles presented a two-phase release profile of the EO. The authors believe that the rapid first phase represents the portion of thymol that was in the external phase of the film; the slower second phase represents thymol that was contained in the zein particles [41].

Polylactic glycolic acid nanocapsules containing eugenol or transcinnamaldehyde both presented a two-phase EO release. The first phase was rapid (under 30 minutes) and approximately 20% of the EO load was detected; the second release phase was prolonged and after 72 hours 64% of eugenol and 87% of transcinnamaldehyde were detected. Considering that PLGA has a low degradation rate, the release was governed mostly by diffusion with a possible influence of polymer swelling and bulk erosion. The first release phase may be attributed to the molecules that are adsorbed to the polymeric wall, while the second release phase represents the EO present in the core of the nanocapsules which diffuses through the polymeric wall [42].

Polylactic glycolic acid nanocapsules containing carvacrol have also been produced. Size was about 209.8 nm, polydispersity was 0.260, zeta potenzial was −18.99, drug loading was 21%, and encapsulation efficiency was 26%.* In vitro* release profile occurred with an initial “burst” release followed by a slower release due to the concentration gradient. Nanoparticles showed a 60% release after 3 h and approach to completeness after 24 h with approximately 95% of carvacrol released. The effect of carvacrol EO antimicrobial activity was enhanced because the nanoparticles significantly altered rheological characteristic of bacterial biofilms potentially facilitating the action of carvacrol [43].

Methyl cellulose/ethyl cellulose polymeric nanoparticles containing thymol attaining the relatively high thymol loading level of 43.53% (weight of encapsulated thymol to weight of the thymol-loaded spheres) were able to reduce and preserve levels of* E. coli* in an oil/water lotion and in a hydrophilic gel, of* P. aeruginosa* in an oil/water lotion and of* S. aureus* in an oil/water lotion and in a water/oil cream. Interestingly, free thymol was also capable of reducing microbiologic levels in these formulations, but the preservation period was shorter except for the* S. aureus* in an oil/water lotion where free thymol maintained low microbial levels for the same period as the nanocapsules. Effective bacterial suppression by encapsulated thymol was also observed when used in cream and aqueous gel formulations [44].

### 5.2. Lipid-Based Nanocarriers

Lipid-based nanocarriers include micro- and nanometric-scaled emulsions and lipid nanoparticles, roughly divided in liposomes, micelles, niosomes, solid lipid nanoparticles (SLN), and nanostructured lipid carriers (NLC). Liposomes and niosomes are colloidal association of amphiphilic lipids that organize themselves spontaneously in bilayer vesicles and that are suitable with hydrophilic and hydrophobic compounds. SLN and NLC are solid particles at room and human body temperatures that present lipid core, which makes these carriers a proper medium for entrapment of lipophilic compounds, as EO.

As these nanoparticles are composed of lipids and/or phospholipids, they have the ability to interact with several cell types. So, these carriers can been seen as alternatives for treatment of microbial infections, due to their capacity of interaction with infected cells. Furthermore, the association of EO with lipid nanoparticles has different objectives, but the main aims are the enhancement of the stability and the solubility in aqueous media of EO, maintenance or even enhancement of their biological activity, and drug targeting.

#### 5.2.1. Micro- and Nanoemulsions

Microemulsions can be defined as homogeneous thermodynamically stable transparent dispersions of two immiscibleliquids stabilized by an interfacial film of surfactants. They have droplet size above 500 nm and require very low energyto formulate emulsion, since they form spontaneously when aqueous, oily, and amphiphilic components are brought intocontact, besides having a lower production cost compared to nanoemulsions. One major drawback to microemulsions isthat formation requires high surfactant concentration, which can cause toxicity when used in pharmaceutical applications.

In contrast nanoemulsions can be prepared using lower surfactant concentrations. Nanoemulsions are fine oil-in-water dispersions, nonequilibrium systems with a spontaneous tendency to separate into the constituent phases. Nevertheless, nanoemulsions may possess a relatively high kinetic stability even for several years, due to their very small size, essentially the consequence of significant steric stabilization between droplets. They have droplet covering the size range of 10–500 nm and also referred to as miniemulsions, ultrafine emulsions, and submicrometer emulsions.

Antimicrobial properties of micro- and nanoemulsion are believed to result from the small size of oil particles that have a high surface tension which can fuse with and subsequently disrupt the membrane of isolated prokaryotic cells, viruses, and eukaryotic cells of fungi but they do not affect eukaryotic cells of higher organisms. A synergistic antimicrobial effect could be afforded by including some substances which possess strong antimicrobial activity into the formula, reducing the amounts of active substances and detergents used for killing microorganisms by the conventional method and the cost of raw materials. Furthermore, irritation caused from detergents in the formula is not likely to happen when they are used in low concentrations.

Encapsulation in nanoemulsion-based delivery systems of two antimicrobial compounds, a terpenes mixture extracted from* Melaleuca alternifolia* and D-limonene, deals with the issues of formulation and fabrication in order to retain and possibly enhance the antimicrobial activity of the encapsulated compounds.

The nanoemulsions based on food-grade ingredients were investigated by determining the minimum inhibitory concentration (MIC) and minimum bactericidal concentration (MBC) for three different classes of microorganisms (*Lactobacillus delbrueckii*,* Saccharomyces cerevisiae*, and* Escherichia coli*). The increase of the antimicrobial activity resulted in dependance on the formulation andmean diameter of the delivery systems as well as on the microorganisms class. Additionally, GC-MS analysis revealed that high intensity processing for nanoemulsion production may affect the chemicalstability of several active compounds.

The results of the accelerated shelf life studies show that for both fruit juices after 2 days, the total inactivation of the initial microbial load of 10^3^ CFU/mL was already reached for the terpenes concentrations of 5.0 g/L and 10 g/L. At a terpenes concentration of 1.0 g/L, microorganism growth is delayed by 5 days in orange juice and 2 days in pear juice in comparison to the control [45].

Another study reported the preparation of a self-nanoemulsifying drug delivery system for the oral delivery of zedoary turmeric oil, an essential oil extracted from the dry rhizome of* Curcuma zedoaria*. The optimized formulation consisting of EO, ethyl oleate, Tween 80, Transcutol P (30.8 : 7.7 : 40.5 : 21, *w*/*w*), and loaded with 30% drug was prepared. Upon mixing with water, the formulation was rapidly dispersed into fine droplets with a mean size of 68.3 ± 1.6 nm and zeta potential of −41.2 ± 1.3 mV. The active components remained stable in the optimized formulation stored at 25°C for at least 12 months. Following oral administration in rats, both AUC and Cmax of germacrone, a representative bioactive marker of zedoary turmeric oil, increased by 1.7-fold and 2.5-fold, respectively, compared with the unformulated zedoary turmeric oil [46].

#### 5.2.2. Liposomes

Liposomes are one of the most studied colloidal delivery systems; in fact, they were first developed for drug delivery purposes as early as 1970s [47, 48].

Liposomes consist of vesicular self-assembled system comprising of one or more bilayers, usually formed using a phospholipid, surrounding an aqueous core. Liposomes can contain (i) one bilayer forming unilamellar vesicles (ULV), (ii) several concentric bilayers forming multilamellar vesicles, or (iii) nonconcentric bilayers forming multivesicular vesicles (MVV). The size of these structures can be rather small (in the range of 20 nm) or rather large (exceeding 1 *μ*m). Owing to the presence of the hydrophilic compartment and lipophilic palisade, they can be used as carriers for both lipophilic and hydrophilic molecules [48].

Bioactive compounds compartmentalised in liposomes can be protected against degradation and in case of lipophilic compounds, liposomal encapsulation can also lead to increased solubilisation [48].

The effect of liposomal inclusion on the stability and* in vitro* antiherpetic activity of* Santolina insularis* EO was investigated. Vesicles were obtained from hydrogenated soya phosphatydilcholine and cholesterol. Formulations were examined for their stability for over one year monitoring the drug leakage from vesicles and the average size distribution. The stability of the incorporated oil was verified by studying its quali-quantitative composition. The antiviral activity was studied against herpes simplex virus type 1 (HSV-1) by plaque reduction and yield reduction assays. Results showed that* Santolina insularis* EO can be incorporated in high amounts in the prepared liposomes, which successfully prevented its degradation. Moreover, stability studies pointed out that vesicle dispersions were stable for at least one year and neither oil leakage nor vesicle size alteration occurred during this period. Antiviral activity assays demonstrated that* Santolina insularis* essential oil is effective in inactivating HSV-1 and that the activity is principally due to direct virucidal effects. Free EO proved to be more effective than liposomal oil and a different activity was discovered which related to the vesicular structure. The ED(50) values, significantly lower when cells were preincubated with the EO before the virus adsorption, indicate an intracellular mechanism in the antiviral activity of* Santolina insularis* [49].

The effect of liposomal inclusion on the* in vitro* antiherpetic activity of* Artemisia arborescens* L. EO was investigated. In order to study the influence of vesicle structure and composition on the antiviral activity of the vesicle-incorporated oil, multilamellar (MLV) and unilamellar (SUV) positively charged liposomes were prepared. Liposomes were obtained from hydrogenated (P90H) and nonhydrogenated (P90) soy phosphatidylcholine. Formulations were examined for their stability for over one year, monitoring the oil leakage from vesicles and the average size distribution. The antiviral activity was studied against herpes simplex virus type 1 (HSV-1) by a quantitative tetrazolium-based colorimetric method. Results showed that* Artemisia* EO can be incorporated in good amounts in the prepared vesicular dispersions. Stability studies pointed out that vesicle dispersions were very stable for at least six months and neither oil leakage nor vesicle size alteration occurred during this period. After one year of storage oil retention was still good, but vesicle fusion was present. Antiviral assays demonstrated that the liposomal incorporation of* A. arborescens* EO enhanced its* in vitro* antiherpetic activity especially when vesicles were made with P90H. On the contrary, no significant difference in antiviral activity was observed between the free and SUV-incorporated oil. P90H MLV showed a higher activity than P90 MLV (EC50 values of 18.3 and 43.6 *μ*g/mL for P90H MLV and P90MLV, resp.), while no significant differences of the antiviral activity were observed between the free essential oil and SUV vesicles. Incorporation of* A. arborescens* essential oil in multilamellar liposomes greatly improved its activity against intracellular HSV-1 [50].

A modified technique of rapid expansion of supercritical solutions (RESS) was applied to incorporate EO extracted from* Atractylodes macrocephala *Koidz into liposomes. The optimised entrapment efficiency, drug loading, and average particle size of liposomes were found to be 82.18%, 5.18%, and 173 nm, respectively. The physicochemical properties including the entrapment efficiency, dissolution rate, and stability met the characteristic for a pharmaceutical use of the developed formulation [51].

Carvacrol, thymol, p-cymene, and c-terpinene were identified as major constituents and isolated from the EOs from* Origanum dictamnus* L. The above components were successfully encapsulated in phosphatidyl choline-based liposomes and the possible improvement of their antioxidant and antimicrobial activities was tested against four Gram-positive and four Gram-negative bacteria and three human pathogenic fungi, as well as the food-borne pathogen,* Listeria monocytogenes*. In order to investigate any possible synergistic or antagonistic effect between carvacrol/thymol and carvacrol/c-terpinene, the antimicrobial activities of the mixtures were also determined before and after encapsulation in liposomes. All tested compounds presented enhanced antimicrobial activities after the encapsulation [52].

A study examined carvacrol (derivatives) and thymol encapsulated in liposomes to increase their bioavailability and stability. Similarly, the endurance to humidity and UV light was enhanced [53].

#### 5.2.3. SLN Solid Lipid Nanoparticles

Solid lipid nanoparticles (SLN) refer to nanoscale size particles prepared using lipids that remain solid at room temperature (or/and body temperature). The lipid component may comprise of a broad range of lipid and lipid-like molecules such as triacylglycerols or waxes [54]. The diameter of such lipid particles can be also quite small, that is, in the range between 50 nm and 1 *μ*m. Active ingredients can be solubilised homogeneously either in the core of the SLNs or in the outside part [55]. The advantage of SLNs as delivery system for lipophilic active components is reported to lie in the immobilisation of active elements by the solid particle structure leading to an increased chemical protection, less leakage, and sustained release [56].

This physical property allows a better control of both the physical (against recrystallisation) and chemical (against degradation) stability of the delivered constituents.

The effect of SLN incorporation on transdermal delivery and* in vitro* antiherpetic activity of* Artemisia arborescens* EO has been investigated. Two different SLN formulations were prepared using the hot-pressure homogenization technique, Compritol 888 ATO as lipid, and Poloxamer 188 (SLN 1) and Miranol Ultra C32 (SLN 2) as surfactants.

One day after production, the SLN 1 had a size of 223 nm (0.243 polydispersion index) while the particle size of SLN 2 prepared using Miranol Ultra C32 as surfactant was 219 nm (0.301 polydispersion index, PI). The mean particle size of the formulations increased only slightly after two years of storage, indicating a high physical stability of both SLN 1 and SLN 2 formulations. In particular, 2 years after production, SLN 1 and SLN 2 formulations showed a mean size of 242 nm (0.285 PI) and 239 nm (0.321 PI). The PI values were always smaller than 0.350 indicating a fairly narrow size distribution of the particles. Formulations were examined for their stability for two years by monitoring average size distribution and zeta potential values. The antiviral activity of free and SLN incorporated EO was tested* in vitro* against Herpes Simplex Virus-1 (HSV-1), while the effects of essential oil incorporation into SLN on both the permeation through and the accumulation into the skin strata were investigated by using* in vitro* diffusion experiments through newborn pig skin and an almond oil* Artemisia essential* oil solution as a control. Results showed that both SLN formulations were able to entrap the EO in high yields and that the mean particle size increased only slightly after two years of storage, indicating a high physical stability.* In vitro* antiviral assays showed that SLN incorporation did not affect the EO antiherpetic activity. The* in vitro* skin permeation experiments demonstrated the capability of SLN of greatly improving the oil accumulation into the skin, while oil permeation occurred only when the oil was delivered from the control solution [57].

Alhaj and coworkers developed a formulation based on* Nigella sativa *essential oil into solid lipid nanoparticles SLN. SLN formulations were prepared using hydrogenated palm oil Softisan 154 and* N*.* sativa *essential oil as lipid matrix, sorbitol, and water. Data showed a high physical stability for formulations at various storage temperatures during 3 months of storage. In particular, average diameter of* N*.* sativa *essential oil loaded SLN did not vary during storage and increased slightly after freeze-drying the SLN dispersions. Therefore, obtained results showed that the studied SLN formulations are suitable carriers in pharmaceutical and cosmetic fields [58].

Frankincense and myrrh are gum resins obtained from the genera* Boswellia *and* Commiphora*, respectively. Both genera belong to the family Burseraceae, which is native to Northeast Africa and the Middle East. Frankincense and myrrh have been used for medical purposes in China and India for thousands of years. Modern pharmacological research has revealed that essential oils are the primary effective components in frankincense and myrrh oil (FMO) that exhibit a broad spectrum of biological activities such as antimicrobial, anti-inflammatory, and antitumor activities. As with other essential oils, the instability and poor water solubility of FMO result in poor oral bioavailability, which limits its clinical application. The components of FMO are sensitive to light, air, and high temperature, and FMO stimulates the gastrointestinal tract, making it unsuitable for oral administration. A study has reported the preparation of solid lipid nanoparticles for the oral delivery of frankincense and myrrh essential oils (FMO). Aqueous dispersions of SLNs were successfully prepared by a high-pressure homogenization method using Compritol 888 ATO as the solid lipid and soybean lecithin and Tween 80 as the surfactants. Round SLNs were with a mean size of 113.3 nm, a zeta potenzial of −16.8 mV, and an encapsulation efficiency of 80.60%. SLN formulation increased the antitumor efficacy of FMO in H22-bearing Kunming mice. Compritol 888 ATO showed reasonable FMO solubilization capacity. The poorly water-soluble drug FMO was efficiently encapsulated into the nanoparticles. Particles prepared under proper formulation conditions were spherical with diameters of 220 nm [59]. Solid lipid nanoparticles (SLNs) of essential oil of* Zataria multiflora* have been developed. The results showed that the encapsulation efficiency was 38.66%. Results of particle size determination showed a mean size of 650 nm and SLNs were spherical as shown by TEM. The DSC curve of sodium dodecyl sulfate, polyethylene glycol, cetyl alcohol, and EO was different from EO containing SLNs, which indicated that the EO can interact with the matrix of lipid during the preparation of the SLNs. 93.2% of the essential oil was released after 24 h. The results of characterization of the SLNs indicated the potential application of essential oil of* Z. multiflora* loaded SLN as carrier system [60].

### 5.3. Molecular Complexes

A simple strategy to deliver active ingredients is by physically complexing them with other molecules in order to have a better solubility profile and/or an increase in the chemical stability of the complexed system. In this context a molecular complex is referring to the physical association between a host and a guest (active ingredient) molecule and in the case of EOs the complexes are reported with cyclodextrins (CDs).

Cyclodextrins are natural macrocyclic oligosaccharides well known for having toroid-shaped structures with rigid lipophilic cavities and a hydrophilic outer surface insuring good dissolution of the complex in an aqueous environment. They are able to enclose highly hydrophobic molecules inside their hydrophobic cavity, constituting a true molecular encapsulation [61]. The major advantages of the use of CD-complexation in pharmaceutical applications, foods, cosmetics, and toiletries are protection of the active ingredients against oxidation, light induced reactions, decomposition and thermal decomposition, loss by evaporation and sublimation, and elimination or reduction of undesired tastes/odours, to reduce or prevent gastric-intestinal irritation (mainly due to anti-inflammatory drugs) or ocular disturbances, prevent drug-drug or drug-additive interactions, or even to convert oils and liquid drugs into microcrystalline or amorphous powders and to reduce microbiological contamination, fibres, or the elimination of other undesired components and hygroscopicity [62]. Moreover, formation of inclusion complex (IC) increases the guest's* in vivo *stability against hydrolysis, oxidation, decomposition, and dehydration, consequently increasing bioavailability and bioefficacy. There are three main types of CDs: *α*-, *β*-, and *γ*-cyclodextrins, corresponding to 6, 7, and 8 glucopyranose units linked by *α*-(1,4) bonds, respectively. The dimensions of the internal cavity are 0.5–0.8 nm and are crucial for the “encapsulation” of guest molecules [63].

In the last years, physicochemical properties and, consequently, the inclusion capacity of the natives' CD have been improved by chemical modification of their hydroxyl groups [64]. Besides natural cyclodextrins, a growing number of semisynthetic derivatives and copolymers have been prepared and are already commercially available. Many of them found use as structural and chiral selectors, with new properties given by the type and number of substituents. The semisynthetic derivatives of cyclodextrins show better solubility in water, can decrease and modulate the release rate of water soluble molecules, are able to enhance the dissolution rate and the inclusion capacity, and also decrease the side effects of some molecules.

The majority of the publications is concerning the encapsulation of essential oils with *β*-CD and its derivatives: randomly methylated-*β*-cyclodextrin, hydroxypropyl-*β*-cyclodextrin, and low methylated-*β*-cyclodextrin.

The IC of thymol and cinnamaldehyde and *β*-CD was investigated [65] in order to study the influence of water adsorption by CDs and their complexes on the release of encapsulated compounds. The results showed that *β*-CD encapsulates efficiently both of them, in a 1 : 1 molar ratio. The ICs were obtained upon mixing the components in aqueous media and subsequent freeze-drying, as confirmed by differential scanning calorimetry. The samples were stored at constant relative humidity, from 22% to 97%, at 25°C. The release of encapsulated compounds was determined following the melting enthalpy of each guest. Water sorption isotherms for *β*-CD and the complexes showed constant and low water sorption at RH < 80%; then the uptake of water increased abruptly. The amount of sorbed water at each RH was smaller for the complexes than for *β*-CD. The guest molecules displaced water molecules from inside the cavity of *β*-CD. No thymol or cinnamaldehyde release was detected at RH < 84%, and it increased abruptly from 84% RH, coincidentally with the abrupt increase of absorbed water. Water sorption significantly affects *β*-CD complexes stability, which is thus governed by the shape of the water sorption isotherm. The stability studies showed that the inclusion complexes thymol-*β*-CD and cinnamaldehyde-*β*-CD remain stable up to 75% RH during long storage times. In fact, the guests released from the *β*-CD complexes were detectable in the region of the water adsorption isotherm at which a sharp increase of water content occurred (84% RH). These results show the relevance of selecting appropriated storage conditions for hydrophobic flavours encapsulated in *β*-CD or for predicting the shelf life of functional products formulated with nanoencapsulated compounds [65].

*β*-Caryophyllene (BCP), a natural sesquiterpene existing in the essential oil of many plants, has exhibited a wide range of biological activities such as antimicrobial, anticarcinogenic, anti-inflammatory, antioxidant, anxiolytic-like, and local anaesthetic effects. However, its volatility and poor water solubility limit its application in pharmaceutical field. Liu and coworkers investigated and compared the oral bioavailability and the pharmacokinetics of free BCP and BCP/*β*-CD IC after a single oral dose of 50 mg/kg on rats [66]. BCP was rapidly released from inclusion complex and the* in vivo* data showed that BCP/*β*-CD IC displayed earlier Tmax, higher Cmax and the AUC0-12 h showed approximately 2.6 times higher increase than those of free BCP. The *β*-CD has significantly increased the oral bioavailability of the drug in rats than free BCP [66].

The essential oil of* Chamomilla recutita* (L.) Rauschert, syn.* Matricaria recutita* L., contains up to 50% (−)-*α*-bisabolol which contributes to the anti-inflammatory properties of camomile oil. Bisabolol is a very lipophilic substance, with a tendency to oxidise decreasing anti-inflammatory activity ca. 50%. (−)-*α*-Bisabolol was found to form an inclusion complex with *β*-CD in solution as well as in the solid state. To investigate molecular associations of *β*-CD with pure (−)-*α*-bisabolol or (−)-*α*-bisabolol as a component of camomile EO, Waleczek et al. undertook phase solubility studies [67]. The complex constant was 273 M^−1^ for the pure (−)-*α*-bisabolol and 304 M^−1^ for (−)-*α*-bisabolol as a constituent of the EO. The intrinsic solubility of pure (−)-*α*-bisabolol (4.85 × 10^−4^ M) and (−)-*α*-bisabolol as a component of the EO (1.82 × 10^−4^ M) differ significantly. Computer simulation proved an inclusion complex having a stoichiometric composition of 2 : 1 (*β*-CD : drug) [67].

Thymol is a monoterpene present in Lamiaceae plants, specially oreganos and thymes. Cinnamaldehyde (3-phenyl-2-propenal) represents 65–75% of the cinnamon EO. Thymol and cinnamaldehyde are frequently used as flavours, but they are also becoming increasingly important as naturally occurring antimicrobial, antioxidant, and antiseptic agents. As natural and artificial flavours they are very sensitive to the effects of light, oxygen, humidity, and high temperatures. The study of Hill et al. [68] aimed to elucidate the physicochemical characteristics of essential oils and *β*-Cyclodextrin (EO-*β*-CD) inclusion complexes and their resulting antimicrobial activity. Cinnamon bark extract, transcinnamaldehyde, clove bud extract, eugenol, and a 2 : 1 (transcinnamaldehyde : eugenol) mixture were microencapsulated by the freeze-drying method. EO-*β*-CD complexes were characterized for particle size, morphology, polydispersity index (PI), entrapment efficiency, and phase solubility. All particles showed a spherical shape, smooth surface, no significant differences in size distribution, and strong tendency to agglomerate. The entrapment efficiencies ranged from 41.7 to 84.7%, where pure compounds were higher (*P* < 0.05) than extracts.

The oils and their *β*-CD complexes were analyzed for their antimicrobial activity against* Salmonella enterica* serovar* Typhimurium* LT2 and* Listeria innocua*. All the samples effectively inhibited bacterial growth within the concentration range tested, except free eugenol. The EO-*β*-CD complexes were able to inhibit both bacterial strains at lower concentrations than free oils, likely due to their increased water solubility which determined an increased contact between pathogens and essential oils. The cinnamon bark and clove bud olis/*β*-CD complexes were the most powerful antimicrobials, despite showing the lowest entrapment efficiencies amongst the oils. The results indicate that such EO inclusion complexes could be useful antimicrobial delivery systems with a broad spectrum of application in food systems where Gram-positive and -negative bacteria could present a risk [68].

Garlic (*Allium sativum* L.) is a widely distributed plant and is used throughout the world not only as a spice and a food, but also as a folk medicine, and many of the beneficial health-related biological effects have been attributed to its characteristic organosulphur compounds [69]. Steam distillation is widely used to extract and condense the volatile organosulphur compounds in garlic, and the final oily product is called garlic oil (GO). The compounds of GO mainly are diallyl disulphide, diallyl trisulphide, allyl propyl disulphide, a small quantity of disulphide, and probably diallyl polysulphide [70]. GO is recognised to be more potent than aqueous extracts of garlic and exhibits a wide range of pharmacological properties including antimicrobial, antidiabetic, antimutagenic, and anticarcinogenic effects [71]. However, the application of GO is limited due to its volatility, strong odour, insolubility in water, and low physicochemical stability.

The characterisation of ICs of GO/*β*-CD was investigated [72]. The calculated apparent stability constant of IC was 1141 M^−1^, and the water solubility of GO was significantly improved. Furthermore, the release rate of GO from the inclusion complex was controlled. The results of this study clearly demonstrated that GO could be efficiently complexed with *β*-CD to form an inclusion complex by the coprecipitation method in a molar ratio of 1 : 1. The aqueous solubility and stability of GO were significantly increased by inclusion in *β*-CD [72].

Isothiocyanates (ITCs) are hydrolysis products of sulphur-containing compounds called glucosinolates, which occur naturally in cruciferous vegetables, such as broccoli and cabbage. Mechanical disruption of cruciferous plant tissues releases ITCs, due to the hydrolysis reaction catalysed by myrosinase bound to the cell wall and possesses antimicrobial activities [73]. ITCs, in particular allyl isothiocyanate (AITC), have been extensively studied for their antibacterial effect for food. Inclusion complexation reactions between isothiocyanates (ITCs), namely, allyl isothiocyanate (AITC) and phenyl isothiocyanate (PITC), and randomly methylated *β*-cyclodextrin (RM-*β*-CD) were reported [74].

The apparent activation energy of IC dissociation suggested a reduction of volatility and physical stabilisation by inclusion complexation.

RM-*β*-CD demonstrated a strong solubilising effect on the poorly water-soluble AITC and PITC in the aqueous phase. RM-*β*-CD was more effective in solubilising PITC though the AITC/RM-*β*-CD complex had higher apparent stability constants. Despite the fact that a greater amount of AITC was solubilised in the aqueous phase at any given concentration of RM-*β*-CD, the solid state AITC/RM-*β*-CD complex showed an inclusion ratio remarkably lower than that of the PITC/RM-*β*-CD complex. Both of the ITCs may form inclusion complexes with RM-*β*-CD at guest to host ratios of 1 : 1 and 1 : 2 in the aqueous phase [74].

The inclusion interactions of cyclodextrins (CDs) and *β*-cyclodextrin polymers with linalool and camphor in* Lavandula angustifolia* EO were investigated in order to prepare novel controlled release systems for the delivery of essential oil used as ambient odours [75].

The complexation behaviour and the retention capacity of *α*-CD, *β*-CD, *γ*-CD, hydroxypropyl-*β*-cyclodextrin (HPBCD), randomly methylated-*β*-cyclodextrin (RAMEB), a low methylated-*β*-cyclodextrin (CRYSMEB), and cross-linked *β*-CD polymers for linalool and camphor, two major components of* Lavandula angustifolia *EO, were studied. The complexation and the retention capacity of CDs and CD polymers were investigated under solid support or in aqueous media by static headspace gas chromatography. The release profile of aroma from solid support was studied by multiple headspace extraction (MHE). The retention capacity of the CD derivatives was measured in static experiments.

The stability constants with monomeric CD derivatives were determined for standard compounds and for the compounds in essential oil. The RAMEB showed the higher formation constant both for the standard compounds (833 M^−1^ for linalool and 1194 M^−1^ for camphor) and for the compounds in the in* Lavandula angustifolia* essential oil (1074 M^−1^ for linalool and 2963 M^−1^ for camphor). All studied CDs and CD polymers reduce the volatility of the aroma compounds and stable 1 : 1 inclusion complexes are formed. *β*-CD is the most versatile CDs for the two guests, leading to greater formation constant and retention ability in aqueous phase [75].

## 6. Concluding Remarks

EOs have promising potentials for maintaining and promoting health, as well as preventing and potentially treating some diseases. However, the generally low water solubility and stability, together with the high volatility and side effects associated with their use have limited their application in medicine. Nanotechnology is an innovative approach that has potential applications in medicinal and health research. Indeed, nanoparticles are a very attractive tool and are able to solve the major inconvenience of EOs use increasing the chemical stability in the presence of air, light, moisture and, high temperatures, factors which can lead to the rapid evaporation and to the degradation of the active components. In addition, nanocarriers ensure the easier and safer handling of the liquid substances by changing them in solid powders, determining retention of volatile ingredients and taste masking, setting up controlled release and/or consecutive delivery of multiple active ingredients, reducing toxic side effects, improving water solubility of hydrophobic ingredients, and enhancing bioavailability and efficacy.

Nanoencapsulation of EOs in liposomes, solid lipid nanoparticles, nano- and microemulsions, and polymeric nanoparticles represent a promising strategy for overcoming EOs limitations, lowering their dose and increasing long-term safety of these constituents.

## Figures and Tables

**Figure 1:** Representative structures typical of essential oils.

**Figure 2:** Skin nanoparticle drug delivery takes place in three major sites: stratum corneum surface through intracellular (2) and intercellular (4) penetration, furrows (1), and openings of hair follicles (3). The nanoparticles are shown in violet.

**Figure 3:** Mechanisms of nanocarriers (violet) enhanced absorption by enteric mucosa.

**Figure 4:** Schematic illustration of nanosystem platforms for essential oils.
